The article "Image Semantic Segmentation Method Based on Deep Fusion Network and Conditional Random Field" was published in 2022. Journal: Comput Intell Neurosci.

# Image Semantic Segmentation Method Based on Deep Fusion Network and Conditional Random Field

**DOI:** 10.1155/2022/8961456

**Published:** 2022-05-14

**Authors:** Shuo Wang, Yi Yang

**Affiliations:** ^1^School of Energy and Intelligence Engineering, Henan University of Animal Husbandry and Economy, Zhengzhou, Henan 450044, China; ^2^School of Information Engineering, Henan University of Animal Husbandry and Economy, Zhengzhou, Henan 450000, China

## Abstract

Aiming at the problems of missing points and wrong points in image semantic segmentation under complex background and small target, an image semantic segmentation method based on the fully convolution neural network and conditional random field is proposed. First, the deconvolution fusion structure is added to the fully convolution neural network to build a deep fusion network. The multiscale features are automatically obtained through the deep fusion network, and the shallow detail information and deep semantic information are fused to improve the processing accuracy of image rough segmentation. Then, the bivariate potential function of the conditional random field is optimized based on the convolution neural network, and it is used for image fine segmentation to obtain the final image segmentation result. Finally, the proposed method is experimentally analyzed based on the Cityscapes dataset. The results show that the proposed method can achieve accurate image segmentation, and the area under the segmentation curve of the overall size target is 93.6%, which is better than other methods.

## 1. Introduction

As an important research direction in the field of computer vision, the ultimate goal of image semantic segmentation is to use the computer to simulate human vision to quickly perceive objects and analyze environmental information, realize image semantic understanding and reasoning, and make corresponding action feedback according to the high-resolution information input by vision [1, 2]. Specifically, image semantic segmentation refers to identifying the specific target and location in the image from the pixel level and depicting the scene contour with different colors through target detection.

At present, semantic segmentation has been widely used in medical images, remote sensing systems, clothing, security, and transportation [3]. In medical image analysis, semantic segmentation is applied to tumor image analysis and tooth lesion judgment [4]. In the satellite remote sensing system, it is used to segment, locate, and label the geographical objects such as roads, rivers, forests, crops, and buildings in the remote sensing image, which can save a lot of manual labeling cost and time cost [5]. In the field of unmanned driving, the vision-based processing method is still an important part, and image semantic segmentation is regarded as an important technology supporting automatic driving application scenarios [6, 7].

The article "Image Semantic Segmentation Method Based on Deep Fusion Network and Conditional Random Field" was published in 2022. Journal: Comput Intell Neurosci.

Although image semantic segmentation has been widely used, there are still some bottlenecks that limit its development. For example, different kinds of objects with similar appearances are difficult to distinguish, and smaller objects are easy to lose details and specific contours, which are all problems to be solved in existing image semantic segmentation [8]. In order to solve these difficulties, most early image semantic segmentation technologies are based on traditional methods, mainly including segmentation methods based on the threshold, edge detection, and region [9]. With the emergence of deep learning, the image semantic segmentation method based on deep learning gradually replaces the traditional methods, and its accuracy, speed, and other performance indicators have been greatly improved [10, 11].

At present, there has been some research on image semantic segmentation in various fields at home and abroad. The traditional image segmentation methods pay more attention to the separation of target and background in the image. There are six traditional image segmentation methods based on the threshold, edge detection, graph theory, region, clustering, and specific theoretical tools. For example, reference [12] analyzed the principles, advantages, and disadvantages of image semantic segmentation based on traditional methods and deep learning methods and pointed out that deep learning network had better optimization results than traditional methods. Reference [13] proposed a new image redirection method using semantic segmentation and pixel fusion, which could finely reassign the scaling factor for each region according to the semantic segmentation results, so as to effectively reduce the geometric distortion in the process of image redirection, but the detection efficiency needs to be improved. Reference [14] proposed an encoder-decoder architecture, which used global and local semantics to solve the problem of automatic image coloring and fine-tune the low-level coding features through scene context classification to integrate the global image style, but it is easy to lose specific details for the contour of small objects. Reference [15] proposed a weak supervision framework for zero sample semantic segmentation, which could segment images with target categories without any pixel-level marker instances, but the effect of image semantic segmentation in a complex environment was poor.

Now, the deep learning algorithm has been widely used in image semantic segmentation [16, 17]. Reference [18] proposed an image semantic segmentation method based on deep learning, which was different from the traditional image segmentation and improved the robustness, timeliness, and accuracy of lane semantic segmentation, but the analysis efficiency and sensitivity of randomly changing images need to be improved. Reference [19] proposed an image semantic segmentation algorithm based on the fully convolution neural network. Reference [20] proposed a crack detection method based on deep learning semantic segmentation. Through the photos of a large number of concrete structures with adverse conditions such as shadow and dirt, the accuracy of the developed method was studied. It was found that not only the crack area could be detected but also the traces of tie rod hole and formwork could be removed, so as to improve the detection accuracy.

The article "Image Semantic Segmentation Method Based on Deep Fusion Network and Conditional Random Field" was published in 2022. Journal: Comput Intell Neurosci.

Based on the above analysis, aiming at the problem of image semantic segmentation with random information in a complex environment, an image semantic segmentation method based on the convolution neural network and conditional random field is proposed. In order to improve the performance of image semantic segmentation, the deconvolution structure is fused into the fully convolution neural network to obtain multiscale features. The shallow detail information and deep semantic information are combined for image rough segmentation, which effectively improves the processing accuracy. The proposed method adopts a fully connected conditional random field model, which can make better use of spatial context information to realize boundary location. The edge contour of the segmented image is clear and close to the label image.

## 2. Image Semantic Segmentation Based on Deep Fusion Network Combined with Conditional Random Field

### 2.1. Algorithm Framework

Before the era of deep learning (DL), the traditional semantic segmentation focuses on the low-order visual information of image pixels [21]. Due to the lack of algorithm training in traditional methods, the algorithm has high complexity, slow convergence, and long time-consuming, and the segmentation effect is often not optimistic. There is no major breakthrough in a long time. With the rapid development of deep learning, breakthroughs have been made in traditional tasks such as image classification. After computer vision entered the era of deep learning, semantic segmentation also begins to try to use the method of deep learning. Semantic segmentation methods based on deep learning continue to emerge, which repeatedly refresh the accuracy of image semantic segmentation.

Aiming at the defects of a large receptive field and weak edge based on a fully convolution network, the proposed method first uses a fully convolution neural network for rough segmentation and then uses a conditional random field for fine segmentation (enhancing edge constraint). Since deep learning, especially convolution neural network, began to be applied to image semantic segmentation, such a general framework has gradually formed, as shown in Figure 1.

The article "Image Semantic Segmentation Method Based on Deep Fusion Network and Conditional Random Field" was published in 2022. Journal: Comput Intell Neurosci.

The front-end image semantic rough segmentation of the network framework is mainly based on the fully convolution network model. The back-end image fine segmentation mostly adopts the undirected probability graph model such as conditional random field, which uses the univariate potential function to describe the information of the current pixel and uses the bivariate potential function to express the information between two pixels. The front-end module is essentially the same as the feature extraction in the traditional method. The back-end module uses the conditional random field to explain the relationship between the essences of transactions and makes pixel-level prediction.

### 2.2. Image Semantic Rough Segmentation Based on Fully Convolution Neural Network

#### 2.2.1. Fully Convolution Neural Network

Since Krizhevsky won the championship in a large-scale image recognition competition by using deep convolution network model, convolution neural network technology has been concerned and applied to related fields by researchers at home and abroad. The advantage of a convolution neural network is that the multilayer structure automatically learns different levels of features. The shallow feature map in the network has richer detailed information. The feature map extracted after multiple convolutions, and pooling operations have deeper semantic information. The fully convolution neural network is mainly composed of four parts: input layer, convolution layer, pooling layer, and output layer.

(1) Input layer: it reads data as an array with dimension *c* × *h* × *d*, where *c* and *h* are sizes of data, and *d* is a feature or channel dimension
(2) Convolution layer: it is also known as the feature extraction layer, which is a process of convolution of input data using filters with specific weights. The features extracted by different convolution kernels are different. The convolution results are output through the activation function. The activation function adopted by the proposed method is rectified linear units (ReLU), which is mathematically expressed as
  (1) $$\begin{array}{c} f\left(x\right)=\max\left(0,x\right). \end{array}$$
(3) Pooling layer: it is also known as the down-sampling layer. In order to avoid the problem of fitting too many parameters, the pooling layer is used to reduce the amount of data and speed up the network training on the basis of retaining useful information. Common pooling operations include maximum pooling and average pooling. The convolution layer and pooling layer can be defined as
  (2) $$\begin{array}{c} y_{ab}=l_{ks}\left({\left(x_{sa+\delta a,sb+\delta b}\right)}_{0\leq \delta a,\delta b<k}\right), \end{array}$$
   where *x*_*ab*_ is the data vector at the position (*a*, *b*), *y*_*ab*_ is the output vector after layer operation (*a*, *b*), *k* is the convolution kernel size, *s* is the step size or down-sampling factor, and *l*_*ks*_ is the type of layer (representing the matrix multiplication or average pooling operation of the convolution layer and the output layer of ReLU function).
(4) Output layer: it outputs the probability vector of each pixel belonging to each semantic category through the Softmax classifier

The article "Image Semantic Segmentation Method Based on Deep Fusion Network and Conditional Random Field" was published in 2022. Journal: Comput Intell Neurosci.

#### 2.2.2. Deconvolution Fusion Structure

The pooling operation in the fully convolution network model training not only reduces the image size but also loses the rich detail information in the image, resulting in low semantic segmentation accuracy [22]. Therefore, deconvolution is used to restore the original image size and realize pixel to pixel image semantic segmentation. At the same time, in order to obtain more accurate semantic segmentation results, the fully convolution network adds a fusion structure, and the shallow detail information in the network model is introduced by combining the pooling layer results of different scales and the final convolution layer results.

*(1) Deconvolution operation*. Deconvolution operation is the operation opposite to convolution operation in the forward and backpropagation of neural network model. Taking the deconvolution operation in the Caffe framework as an example, first, the forward and backpropagation process of convolution operation is analyzed. The forward propagation process is as follows:

(3) $$\begin{array}{c} O=\kappa \times F, \end{array}$$

where *κ* is the convolution kernel matrix, *F* is the image feature matrix, and *O* is the output matrix. During backpropagation, according to the matrix differential formula,

(4) $$\begin{array}{c} \frac{\partial Mx+z}{\partial x}=M^{T}, \end{array}$$

where *M* represents arbitrary matrix, *M*^*T*^ is the transpose matrix of *M*, and *z* is arbitrary constant. It can be deduced as

(5) $$\begin{array}{c} \frac{\partial \text{Loss}}{\partial F}=\frac{\partial \text{Loss}}{\partial O}\cdot \frac{\partial O}{\partial F}=\kappa^{T}\frac{\partial \text{Loss}}{\partial O}, \end{array}$$

where Loss is the loss function, and *κ*^*T*^ is the transpose matrix of *κ*. Therefore, deconvolution is the operation of left multiplication *κ*^*T*^ in forward propagation and left multiplication (*κ*^*T*^)^*T*^ in reverse.

*(2) Fusion structure*. In order to make full use of the detailed information of the image, a fusion structure combining shallow detail information and deep semantic information is adopted. The deep fusion network (DFN) model is shown in Figure 2. The fusion structure is mainly composed of a convolution layer, deconvolution layer, and bonding layer, in which the results from different layers are summed and output. The final convolution layer result of the fully convolution network model only contains the information of the last pooling layer. The model obtained by directly deconvoluting this result is called DFN-5. According to the different depths of the combined pooling layer, it is recorded as models DFN-4, DFN-3, DFN-2, and DFN-1, which respectively represent the depth of the combined pooling layer to pool4, pool3, pool2, and pool1.

The article "Image Semantic Segmentation Method Based on Deep Fusion Network and Conditional Random Field" was published in 2022. Journal: Comput Intell Neurosci.

Taking DFN-4 as an example, the fusion structure deconvolutes the result of the last convolution layer to the output size of pool4 layer and outputs the result after convolution with pool4 layer through the combination layer. Then, it deconvolutes the result of the combination layer to the input image size and obtains the final semantic segmentation result by using the Softmax classifier. The model DFN-3 deconvolutes the results of the combination layer in DFN-4 to the output size of the pool3 layer, outputs the results after convolution with the pool3 layer through the combination layer, and then deconvolutes the results of the combination layer to the input image size for Softmax classification. Models DFN-2 and DFN-1 follow the same process.

In the adopted DFN model, the pooling layers are pool1, pool2, pool3, pool4, and pool5 from left to right. The step size of all convolution layers is 1. The size of the pooling layer kernel is 2, and the step size is 2. The deconvolution step size is half of the deconvolution kernel size. Aiming at the defects of large segmentation receptive field and the weak edge of the fully convolution network, the proposed method introduces context information with the help of the second-order potential function of a conditional random field, fully considers the relationship between pixels, improves the accuracy of semantic segmentation, and refines the edge of semantic segmentation results.

### 2.3. Image Semantic Segmentation Based on Conditional Random Field

A conditional random field is applied to image semantic segmentation. Each image is represented by an undirected graph. Each pixel corresponds to the vertex in the undirected graph, and the connection relationship between pixels corresponds to the connecting lines of the vertex in the undirected graph [23, 24]. In the process of image semantic segmentation, different semantic labels are assigned to each pixel. Two pixels with similar location and color features are more likely to be assigned the same semantic label and less likely to be segmented, which corresponds to the probability model in a conditional random field.

The article "Image Semantic Segmentation Method Based on Deep Fusion Network and Conditional Random Field" was published in 2022. Journal: Comput Intell Neurosci.

Assuming that in the input image, the semantic label of each pixel is expressed as *X*, the predicted value matched with the pixel is expressed as *Y*, the pixel corresponds to the vertex in the graph, and the association between pixels corresponds to the edge in the graph, so the image can be processed by conditional random field. In a conditional random field, there are usually two potential functions. The information of each pixel in the image can be expressed by a univariate term, and the correlation between two pixels in the image can be expressed by a bivariate term. In principle, pixels with similar distances will be assigned the same semantic labels as much as possible, and pixels with obvious differences need to be assigned different labels. The evaluation index of “distance” defined by color difference and spatial relative distance ensures that the image can be accurately cut at the edge with a large gradient to a certain extent [25, 26]. Different from the ordinary conditional random field, the bivariate term in the fully connected conditional random field expresses the correlation between each pixel and all other pixels in the image.

In the proposed method, the image semantic fine segmentation module adopts the fully connected conditional random field model, which is an undirected graph model. The vertices in the graph match the pixels in the image, and the edges in the graph match the association between the pixels in the image. The energy function of the model is as follows:

(6) $$\begin{array}{c} E\left(Y\right)=\sum_{\forall i\in v}\phi \left(Y_{i}^{u}\right)+\sum_{\forall i,j\in \varpi }\psi \left(Y_{i}^{u},Y_{j}^{v}\right), \end{array}$$

where *Y*_*i*_^*u*^ ∈ {0,1} represents whether the pixel *i* has a label *u*. ∀*u* ∈ *L* represents a set of a label *L*; *Y*, *v*, *ϖ* represent a set of potential variables, node sets, and edge sets, respectively; *ϕ*(*Y*_*i*_^*u*^) is a univariate potential function used to measure the cost of assigning the category label *u* to the pixel *i*. For example, if the pixel *i* belongs to the first category label rather than the second category label, *ϕ*(*Y*_*i*_^1^ < *Y*_*i*_^2^) can be obtained; *ψ*(*Y*_*i*_^*u*^, *Y*_*j*_^*v*^) is a bivariate potential function, which is used to measure the penalty of assigning labels *u* and *v* to pixels *i* and *j*.

The article "Image Semantic Segmentation Method Based on Deep Fusion Network and Conditional Random Field" was published in 2022. Journal: Comput Intell Neurosci.

The univariate potential function represents the classification of each pixel, and the bivariate potential function represents a set of smoothing constraints. *ϕ*(*Y*_*i*_^*u*^) is usually defined as

(7) $$\begin{array}{c} \phi \left(Y_{i}^{u}\right)=-\ln\;P\left(Y_{i}^{u=1}=1|I\right), \end{array}$$

where *P*(*Y*_*i*_^*u*^=1*|I*) represents the probability that the pixel *i* belongs to the category label *u*; *I* is the pixel position coordinate. The smooth bivariate term is usually defined as

(8) $$\begin{array}{c} \psi \left(Y_{i}^{u},Y_{j}^{v}\right)=\lambda \left(u,v\right)D\left(i,j\right), \end{array}$$

where *λ*(*u*, *v*) represents the penalty when any pair of labels appear globally at the same time. For example, when the label *u* and *v* do not exist at the same time, the output value should be very large; *D*(*i*, *j*) is the distance between pixels, which is defined as *D*(*i*, *j*)=*ω*_1_‖*I*_*i*_ − *I*_*j*_‖^2^+*ω*_2_‖[*X*_*i*_*Y*_*i*_] − [*X*_*j*_*Y*_*j*_]‖^2^, where *I*_*i*_ represents a feature vector, such as the RGB value extracted from the pixel *i*, Xi and Yi represent the coordinates of the pixel positions, *ω*_1_ and *ω*_2_ represent the constant terms. If two pixels are close and look similar, they tend to have consistent labels.

However, the choice of such a bivariate potential function model has the following two defects: (1) although the first term of the bivariate potential function can capture the consistency frequency between two labels in the training data, it ignores the spatial context between objects. For example, people may appear next to the table, but they will not appear at the bottom of the table. This spatial context relationship is a fusion of patterns; that is, there are different configurations of the positional relationship between objects in different images. (2) It only defines the pairwise relationship between pixels but ignores the high-level semantic interaction between them.

In order to solve these two problems, the proposed method uses the output result based on the fully convolution neural network as the univariate potential function of the fully connected conditional random field, and the original bivariate potential function model is replaced by the following formula:

(9) $$\begin{array}{c} \psi \left(Y_{i}^{u},Y_{j}^{v}\right)=\sum_{q=1}^{Q}\gamma_{q}u_{q}\left(i,u,j,v\right)\sum_{\forall v\in N_{j}}D\left(j,z\right)P_{w}^{v}, \end{array}$$

where ∑_*q*=1_^*Q*^*γ*_*q*_*u*_*q*_(*i*, *u*, *j*, *v*) represents the fusion of local label context, as the punishment for giving labels in the local area, in which *Q* represents the number of different parts in the fusion; *γ*_*q*_ is an indicator variable, similar to a Boolean value, indicating which part is activated and defined as *γ*_*q*_ ∈ {0,1}, and ∑_*q*=1_^*Q*^*γ*_*q*_=1. A more intuitive expression is as follows: pixel *j* is the adjacent pixel of pixel *i*; that is, *j* ∈ *N*_*i*_. (*i*, *u*) represents that the pixel *i* is assigned as the label *u*. *λ*(*i*, *u*, *j*, *v*) is the label cost based on the relative position relationship between (*i*, *u*) and (*j*, *v*). For example, if two labels represent “person” and “table”, and the pixel of “person” is located at the lower part of the pixel of “table”, the value of the learned penalty function should be large. ∑_∀*v*∈*N*_*j*__*D*(*j*, *w*)*P*_*w*_^*v*^ basically simulates a penalty function term involving three pixels: *i*, *j*, and the adjacent points of *j*. If (*i*, *u*) and (*j*, *v*) are consistent, (*i*, *u*) should be consistent with the adjacent pixel (*w*, *v*),  ∀ *w* ∈ *N*_*j*_ of the pixel *j*.

The article "Image Semantic Segmentation Method Based on Deep Fusion Network and Conditional Random Field" was published in 2022. Journal: Comput Intell Neurosci.

### 2.4. Auxiliary Loss

There are many branches in the proposed network, and the learning contents of each branch are different. In order to better supervise the training process of each branch, the auxiliary loss is added to the network during training [27]. In the auxiliary loss, first, through convolution, batch standardization, ReLU, the feature map is obtained, and the number of channels is the same as the number of categories. Unlike the feature fusion module, because it is the final output result, the feature map is upsampled to the input size by bilinear interpolation, and finally, the loss is calculated.

## 3. Experiment and Analysis

In the experiment, Cityscapes dataset is used for analysis and demonstration. Cityscapes is a dataset focusing on the understanding of urban street scenes. Cityscapes contains 30 categories (the actual label range is 0–33, i e., 34 categories), of which 19 classes are used for segmentation tasks. The data are collected during the day, and the sampling conditions are diverse, covering three different seasons of spring, summer, and autumn and different weather conditions (excluding extreme weather environments). The data contain a large number of small objects, the scene scale is changeable, and the background is complex. The dataset contains a total of 5000 images with fine annotation information and 20000 images with rough marks, which are not commonly used. In the semantic segmentation task, only 5000 images with fine annotation are generally used, including 2800 images for training, 600 images for validation, and 1600 test images. The test set label is also confidential and can only be tested by submitting the results to the server of the dataset. It is worth noting that the images in the dataset have a high resolution of 2048×1024. The segmentation examples of the Cityscapes dataset are shown in Figure 3.

The article "Image Semantic Segmentation Method Based on Deep Fusion Network and Conditional Random Field" was published in 2022. Journal: Comput Intell Neurosci.

### 3.1. Evaluation Index

When evaluating the proposed segmentation method, the Precision and Recall of the prediction results are calculated to measure the target classification ability and target detection ability of the model. In addition, by setting different confidence thresholds, the Precision-Recall curve of the model, that is, the P-R curve, is drawn to intuitively show the segmentation effect of the model. When calculating the Precision and Recall indicators of the model, first of all, the test results need to be divided into four categories according to the real label: true positive(TP), true negative (TN), false positive (FP), and false negative (FN).

Precision is obtained by calculating the proportion of correctly predicted samples to all predicted samples in the test results, that is, the proportion of the number of correctly detected samples in the total detected samples, which can reflect the classification ability of the model to the target. The formula of Precision is

(10) $$\begin{array}{c} \text{Precision}=\frac{\text{TP}}{\text{TP}+\text{FP}}. \end{array}$$

Recall is obtained by calculating the proportion of the number of correctly predicted samples to all the real samples in the test results, that is, the proportion of the number of correctly detected samples to the number of real samples, which can reflect the detection ability of the model to the target. The formula of Recall is

(11) $$\begin{array}{c} \text{Recall}=\frac{\text{TP}}{\text{TP}+\text{FN}}. \end{array}$$

Because the two indicators of Precision and Recall are contradictory, the fixed intersection over union (IOU) threshold and confidence threshold are used to judge whether the detection result is correct. When the IOU threshold and object confidence threshold are high, the calculated Precision value is high, and the Recall value is low. Therefore, in order to comprehensively compare the network performance, it is compared through the P-R curve. The P-R curve takes Precision as the abscissa and Recall as the ordinate. The larger the area surrounded under the curve, the better the performance of the model.

### 3.2. P-R Curve Compared with Other Methods

In order to compare the detection performance of the proposed method with other mainstream methods on objects with different scales, in the experiment, the object is set with the scale of [0,64] pixels as the small target, the object with the scale of [64,192] pixels as the middle target, and the object with the scale of [192, 500] pixels as the large target. Then, the confidence level is adjusted, and the Precision and Recall values of prediction results of the model in small target, medium target, large target, and the target with overall scale [0, 500] pixels are calculated, respectively. The P-R curve is shown in Figure 4.

The article "Image Semantic Segmentation Method Based on Deep Fusion Network and Conditional Random Field" was published in 2022. Journal: Comput Intell Neurosci.

It can be seen from Figure 4 that the P-R curve of the proposed method can largely surround the P-R curve of the methods in reference [15] and reference [20] in the detection results of objects with different scales, which shows that the detection of objects with various scales is improved in varying degrees by combining fully convolution neural network and conditional random field. Reference [15] proposes a weak supervision method for zero sample semantic segmentation, which can complete image segmentation without any pixel-level marker instances, but the segmentation effect is poor for most complex environments. Reference [20] proposes a semantic segmentation method based on deep learning, which can realize the image segmentation of small cracks. Therefore, the segmentation effect in [0,64] pixels is not different from that of the proposed method. However, with the increase of pixels, the single segmentation algorithm in reference [20] can not process a large number of images, so the segmentation effect decreases.

### 3.3. Comparison of Visual Segmentation Results

The visual comparison results between the proposed method and the methods in reference [15, 20] on the Cityscapes validation dataset are shown in Figure 5, in which some areas with obvious differences are marked with red dashed boxes.

From the area marked by the red dashed box, it can be seen that the segmentation performance of the proposed method is better than other comparison methods in the details of the Cityscapes validation dataset. First, look at the list of images on the left and their segmentation results. The front wheel of the bike marked with the red dashed box is partially interspersed with the lamppost. Both the methods in reference [20] and the proposed methods are effective in completely identifying the front wheel of the bike and ignoring the lamppost behind. In the right column of pictures, it can be seen from the red dashed box that the segmentation results of reference [15] mistakenly identify the similar signs on the wall as traffic warning signs, and the results of the method in reference [20] are consistent with the results of the proposed method. Of course, there is still a certain gap between the segmentation results of the methods in reference [15, 20] and the proposed methods. There are still deficiencies in the processing of some details, which need to be improved.

The article "Image Semantic Segmentation Method Based on Deep Fusion Network and Conditional Random Field" was published in 2022. Journal: Comput Intell Neurosci.

It should be noted that in the image segmented by the proposed method, there are some scattered black areas, while the color images displayed by other methods have no black areas. This is because, in the annotation of the proposed method, the black areas represent the negligible parts, and the objects in this part are not added to the semantic segmentation task, which belongs to the object category other than the 19 categories in the dataset. In general, the results on the Cityscapes dataset show that the proposed method adaptively enhances the semantic information of low-level features and obtains better segmentation results through the combination of rough segmentation and fine segmentation.

### 3.4. AUC Comparison of Several Detection Methods

In order to compare the detection performance of the three detection methods on various scales numerically, the area under curve (AUC) enclosed by each curve and coordinate axis is calculated, and the calculation results are shown in Table 1.

As can be seen from Table 1, the detection performance of the three methods for medium-sized targets is better than that for small targets and large targets, which is due to the fact that the medium-sized targets in the Cityscapes dataset occupy most of the samples. In addition, the detection results of the proposed method on all scales are better than the other two detection methods, and the AUC of overall size target segmentation is 93.6%. Moreover, compared with reference [20], target detection results are improved by up to 5.4%, indicating that the combination of the fully convolution neural network and conditional random field for rough and fine image segmentation can alleviate the multiscale problem in the target detection method. At the same time, compared with reference [15], the AUC of the proposed method in the segmentation of overall size targets is improved by 7.1%, and the segmentation effect is remarkable.

## 4. Conclusion

At present, most of the existing image segmentation researches focus on integrating feature information of different depths to improve the performance of segmentation tasks. Some of them strengthen the features before feature fusion but focus on the overall enhancement of features and ignore the local differences of features. Therefore, an image semantic segmentation method based on the fully convolution neural network and conditional random field is proposed. Among them, the rough segmentation result of the image is obtained by DFN, which is taken as the first-order potential of the fully connected conditional random field. The spatial context information is introduced through the Gaussian second-order potential function to realize the fine segmentation of the image. The experimental results based on the Cityscapes dataset show that the proposed method can obtain multiscale features with the help of DFN, so its P-R curves are ideal under different pixels. Combined with the image fine segmentation results obtained by conditional random field, the AUC of the overall size target is 93.6%, and the segmentation results are more accurate.

The article "Image Semantic Segmentation Method Based on Deep Fusion Network and Conditional Random Field" was published in 2022. Journal: Comput Intell Neurosci.

The proposed method focuses on the improvement of accuracy without considering the real time. Although many researchers have invested in the research of real-time image semantic segmentation, it still needs to be deeply explored from the practical application to ensure the reliability of recognition results and the security of the application. For example, in the automatic driving scene, not only the accuracy of the model and high recognition speed are required but also the application safety is still a major factor worthy of consideration.

## Figures and Tables

**Figure 1:** Framework of image semantic segmentation network.

**Figure 2:** Deep fusion network model.

**Figure 3:** Segmentation examples of Cityscapes dataset.

**Figure 4:** Comparison of P-R curves between the proposed method and other methods. (a) The target scale is [0, 64] pixels. (b) The target scale is [64,192] pixels. (c) The target scale is [192, 500] pixels. (d) The target scale is [0, 500] pixels.

**Figure 5:** Comparison of visual segmentation results on Cityscapes dataset.

**Table 1:** AUC comparison of three methods.

Method	Ref. [15]	Ref. [20]	Proposed method
Small target	0.836	0.878	0.902
Medium target	0.871	0.903	0.957
Big target	0.908	0.896	0.949
Overall scale target	0.865	0.884	0.936

## Data Availability

The data used to support the findings of this study are included within the article.

## References

[1] Liu W. (2021). Real-time obstacle detection based on image semantic segmentation and fusion network. *Traitement du Signal*.

[2] Xu C.-H., Shi C., Chen Y.-N. (2021). End-to-end dilated convolution network for document image semantic segmentation. *Journal of Central South University*.

[3] Mi L., Chen Z. (2020). Corrigendum to “Superpixel-enhanced deep neural forest for remote sensing image semantic segmentation. *ISPRS Journal of Photogrammetry and Remote Sensing*.

[4] Mi L., Chen Z. (2020). Superpixel-enhanced deep neural forest for remote sensing image semantic segmentation. *ISPRS Journal of Photogrammetry and Remote Sensing*.

[5] Li Y., Shi T., Zhang Y., Chen W. Z. H. (2021). Learning deep semantic segmentation network under multiple weakly-supervised constraints for cross-domain remote sensing image semantic segmentation. *ISPRS Journal of Photogrammetry and Remote Sensing*.

The article "Image Semantic Segmentation Method Based on Deep Fusion Network and Conditional Random Field" was published in 2022. Journal: Comput Intell Neurosci.

[6] Qian G. A., Qd A. (2021). Semantic image segmentation based on SegNetWithCRFs. *Procedia Computer Science*.

[7] Zhu S. (2021). Semantic segmentation of remote sensing image based on convolutional neural network. *Computer Science and Application*.

[8] Zhu Y., Zhao M. (2021). Registration of laser point cloud and optical image in urban area based on semantic segmentation. *Acta Photonica Sinica*.

[9] Mamoon S., Manzoor M. A., Zhang F. E., Ali Z. J.-f. (2020). SPSSNet: a real-time network for image semantic segmentation. *Frontiers of Information Technology & Electronic Engineering*.

[10] Rezaei M., Yang H., Meinel C. (2020). Recurrent generative adversarial network for learning imbalanced medical image semantic segmentation. *Multimedia Tools and Applications*.

[11] Khan M. Z., Gajendran M. K., Lee Y., Khan M. A. (2021). Deep neural architectures for medical image semantic segmentation: review. *IEEE Access*.

[12] Oluwasammi A., Aftab M U., Qin Z., Ngo S T (2021). Features to text: a comprehensive survey of deep learning on semantic segmentation and image captioning. *Complexity*.

[13] Yan B., Niu X., Bare B., Tan W. (2020). Semantic segmentation guided pixel fusion for image retargeting. *IEEE Transactions on Multimedia*.

[14] Nguyen-Quynh T.-T., Kim S.-H., Do N.-T. (2020). Image colorization using the global scene-context style and pixel-wise semantic segmentation. *IEEE Access*.

[15] Shen F., Wang Z. H., Lu Z. M. (2020). Weakly supervised classification model for zero‐shot semantic segmentation. *Electronics Letters*.

[16] Niu X., Yan B., Tan W., Wang J. (2020). Effective image restoration for semantic segmentation. *Neurocomputing*.

[17] Liu K., Ye Z., Guo H., Cao D. L. F.-Y. (2021). FISS gan: a generative adversarial network for foggy image semantic segmentation. *IEEE/CAA Journal of Automatica Sinica*.

[18] Weiwei C. W., Wang K., Wang K., Li Z., Li H., Liu S. (2020). Lane departure warning systems and lane line detection methods based on image processing and semantic segmentation: a review. *Journal of Traffic and Transportation Engineering*.

[19] Choi J., Choi B. (2021). Highly contrast image correction for dim boundary separation of image semantic segmentation. *IEEE Access*.

[20] Yamane T., Chun P.-j. (2020). Crack detection from a concrete surface image based on semantic segmentation using deep learning. *Journal of Advanced Concrete Technology*.

[21] Fan J., Zhang Z., Tan T., Song C. J. (2020). CIAN: cross-image affinity net for weakly supervised semantic segmentation. *Proceedings of the AAAI Conference on Artificial Intelligence*.

The article "Image Semantic Segmentation Method Based on Deep Fusion Network and Conditional Random Field" was published in 2022. Journal: Comput Intell Neurosci.

[22] Wu T., Tang S., Zhang R., Cao J. Y. (2021). CGNet: a light-weight context guided network for semantic segmentation. *IEEE Transactions on Image Processing*.

[23] Ding H., Jiang X., Shuai B., Liu A. Q. G. (2020). Semantic segmentation with context encoding and multi-path decoding. *IEEE Transactions on Image Processing*.

[24] Shimoda W., Yanai K. (2020). Weakly supervised semantic segmentation using distinct class specific saliency maps. *Computer Vision and Image Understanding*.

[25] Zhao S., Hao G., Zhang Y., Wang S. (2021). A real-time semantic segmentation method of sheep carcass images based on ICNet. *Journal of Robotics*.

[26] Zhang L., Hu X., Zhou Y., Zhou G. S. (2021). Memristive DeepLab: a hardware friendly deep CNN for semantic segmentation. *Neurocomputing*.

[27] Kotaridis I., Lazaridou M. (2021). Remote sensing image segmentation advances: a meta-analysis. *ISPRS Journal of Photogrammetry and Remote Sensing*.

